The article "Polymerase Spiral Reaction (PSR): A novel isothermal nucleic acid amplification method" was retracted in 2023. Reasons: errors in the data; errors in the analysis; errors in the methods; unreliable results or conclusions.

# Polymerase Spiral Reaction (PSR): A novel isothermal nucleic acid amplification method

**DOI:** 10.1038/srep12723

**Published:** 2015-07-29

**Authors:** Wei Liu, Derong Dong, Zhan Yang, Dayang Zou, Zeliang Chen, Jing Yuan, Liuyu Huang

**Affiliations:** 1 Institute of Disease Control and Prevention, Academy of Military Medical Sciences, Beijing, 100071, China

## Abstract

In this study, we report a novel isothermal nucleic acid amplification method only requires one pair of primers and one enzyme, termed Polymerase Spiral Reaction (PSR) with high specificity, efficiency, and rapidity under isothermal condition. The recombinant plasmid of *bla*_NDM-1_ was imported to *Escherichia coli* BL21, and selected as the microbial target. PSR method employs a *Bst* DNA polymerase and a pair of primers designed targeting the *bla*_NDM-1_ gene sequence. The forward and reverse Tab primer sequences are reverse to each other at their 5’ end (Nr and N), whereas their 3’ end sequences are complementary to their respective target nucleic acid sequences. The PSR method was performed at a constant temperature 61 °C–65 °C, yielding a complicated spiral structure. PSR assay was monitored continuously in a real-time turbidimeter instrument or visually detected with the aid of a fluorescent dye (SYBR Greenı), and could be finished within 1 h with a high accumulation of 10^9^ copies of the target and a fine sensitivity of 6 CFU per reaction. Clinical evaluation was also conducted using PSR, showing high specificity of this method. The PSR technique provides a convenient and cost-effective alternative for clinical screening, on-site diagnosis and primary quarantine purposes.

Nucleic acid amplification technology has been greatly developed since the invention of polymerase chain reaction (PCR)^1^. PCR has become one of the most valuable tools in virtually all life science fields and significantly promoted the process of molecular biology. However, PCR and its derivatives (such as real-time PCR and Nested PCR) could not get rid of the restriction of thermal cycling for heating and cooling^2^,^3^,^4^.

A wide variety of isothermal amplification techniques have been reported for amplification of DNA or RNA in the past 20 years, including Transcription-based amplification system (TAS)^5^, Self-sustained sequence replication reaction (3SR)^6^, Nucleic acid sequence-based amplification (NASBA)^7^, Strand displacement amplification (SDA)^8^, Rolling circle replication (RCR)^9^, Loop-mediated isothermal amplification (LAMP)^10^, Helicase-dependent amplification (HDA)^11^, Single primer isothermal amplification (SPIA)^12^ and cross-priming amplification (CPA)^13^. Within these methods, TAS, 3SR, NASBA, SDA, HDA and SPIA require multiple enzymes (three or more) and rigorous optimization. Only a few of these isothermal amplification methods (e.g., RCR, LAMP and CPA) can be efficiently performed at a constant temperature using one enzyme. However, RCR method can only amplify circular DNA while four or more primers are indispensable to initiate a LAMP or CPA reaction.

In this study, we describe a novel isothermal nucleic acid amplification method, named Polymerase Spiral Reaction (PSR). Only one pair of primers and one enzyme are needed to launch the PSR reaction, just like PCR. Besides, since the reaction is performed at a constant temperature, an energy intensive thermal cycler is not needed. Moreover, the positive results could be determined through a visual color change. The PSR method is appropriate for on-site and point of care testing.

The main objective of the present study was to demonstrate an application of the PSR method. We chose the *bla*_NDM-1_ gene as the model target. It is a super antibiotic resistance gene emerged in recent years^14^.

## Results

### Characterization of PSR Assay

Like many other isothermal amplification methods, the PSR method relies on the utilization of a DNA polymerase with strand displacement activity. Two primers with reverse sequences at their 5’ end are indispensable to initiate the reaction.

As shown in Fig. 1, primers for the PSR assay, including the forward primer (Ft) and the backward primer (Bt), were designed to target the *bla*_NDM-1_ gene. The uppercase 3’ sequences of the forward primer (F) and reverse primer (B) are complementary to the target *bla*_NDM-1_ gene sequence (position 32922–32941, 33115–33097, GenBank accession: 11027496). The lowercase 5’ sequence of the forward primer (Nr) is reverse to the lowercase 5’ sequence of the reverse primer (N). Nr and N sequences were abstracted from a botanic gene.

The mechanism of PSR method is illustrated in Fig. 1A. When the temperature reaches 61–65 °C, the double-stranded structure of template DNA unlocks due to the presence of Betaine. In the left diagram, F segment of the Ft primer anneals to one single-stranded DNA and extends (structure 1 to structure 2). After the melting of structure 2, the B segment of the Bt primer hybridizes to it (structure 3) and extends (structure 4). The double strands of structure 4 melts and forms a single chain (structure 5). Sequence Nr and N are reverse to each other, and sequence Nr and Nrc are complementary to each other. Thus, sequence N and Nrc are reverse and complementary to each other. Structure 5 would curl to structure 6. The 3’ end of Nrc would continue to extend and finally forms a spiral structure (structure 7). Similarly, the extension mechanism of another single-stranded chain in the right diagram is the same as the left diagram.

Genomic DNA was extracted from 6 × 10^6^ *E. coli* pGEX-NDM-BL21 CFU. A 10-fold DNA dilution series using sterilized double-distilled water resulted in 6000, 600, 60, 6, 0.6 and 0.06 CFU per reaction was used to evaluate the sensitivity of the PSR assay. As depicted in Fig. 2A, samples of genomic DNA extracted from 6000, 600 and 60 CFU were amplified by PSR method within 31 minutes, and the crossing threshold (Ct) value of 6 CFU sample was about 39 min. The 0.6, 0.06 CFU/reaction templates were negative for amplification, as well as the negative control (double-distilled water). Therefore, the sensitivity of PSR method for *E. coli* pGEX-NDM-BL21 containing *bla*_NDM-1_ gene is 6 CFU per reaction. Meanwhile, the standard curve obtained by plotting the value of Ct versus the concentration of CFU (Fig. 2B) shows a fine regression coefficient (R^2^ = 0.9989).

The PSR assay products for the sensitivity test were separated by 1% agarose gel (Armesco) electrophoresis and stained with GelRed (Biotium). Images were documented with a Gel Doc EQ imaging system (Bio-Rad). A typical positive PSR assay produced a ladder of multiple bands on an agarose gel (Fig. 3A, lane 1–4), suggesting that DNA with repeat target sequences were produced due to different spiral amplification stages as a result of simultaneous *Bst* DNA polymerase extension at 3’ end and strand displacement at 5’ end.

SYBR Greenı can bind to double-stranded DNA, emitting green fluorescence under UV light. Experiments were also performed to determine the detection limit of *bla*_NDM-1_ PSR assay when SYBR Greenı was used to enable observation of positive reactions using a visual color change instead of turbidity detection. The PSR assay was performed as described above in a temperature constant water bath. After the termination of reaction, 1 μl of 1:20 diluted SYBR Greenı (Life technologies) was added to the PSR products. The color change could be observed by the naked eye under natural light or under UV light at 365 nm. As shown in Fig. 3B, one minute after the addition of SYBR Greenı, tubes 1 to 4 turned green (positive), and 5 to 7 remained light orange (negative), which was consistent with the real-time assay and the gel electrophoresis result.

To analyze the PSR reaction product, the product was purified with a DNA purification kit (Tiangen Co. China), and digested with Taq I and Hinf I, two restriction enzyme cutting sites found in the original sequence (Fig. 1B). The result showed that the product was digested and formed a single fragment (Fig. 4, Lane 1, 3). Furthermore, two bands in lane 2 (Fig. 4) were excised from the gel, ligated into a TA vector and sequenced. The sequences obtained corresponded to the predicted PSR product of *bla*_NDM-1_ sequence.

### Clinical evaluation of PSR assay

Specificity test and application to clinical diagnosis are also important issues in any diagnostic laboratory. We evaluated the specificity of PSR assay for detecting *bla*_NDM-1_ gene by assessing its reactivity with clinical bacterial strains without *bla*_NDM-1_ isolated in our microorganism center (Table 1)^15^. We observed that the increased turbidity curve appeared only when strains with *bla*_NDM-1_ were used as the template, while the other strains, including the blank control, were negative for amplification (Fig. 5A). Results of traditional PCR (Fig. 5B) and visual test (Fig. 5C) corresponded with the real-time assay, indicating that PSR was specific to *bla*_NDM-1_.

The PSR method was also applied to a clinical screening. 78 clinical sputum samples were collected for PSR-based surveillance of *bla*_NDM-1_ from ICU patients with clinically suspected multi-resistant infections in three top hospitals of Beijing. Ten sputum samples from healthy people were collected as controls. Both PSR and PCR assay were involved to analyze the clinical samples. Of the 78 clinical samples, PSR detected 4 positive samples, which was consistent with PCR assay. Then, the species identification was performed using an automated system (Phoenix and BD systems). Three *Acinetobacter baumannii* strains and one *Klebsiella pneumoniae* strain harboring *bla*_NDM-1_ were successfully cultured from these positive samples. Control samples from healthy people all tested negative in each of the assays. The sequence analysis of the *bla*_NDM-1_ gene from these isolates confirmed conservation with the nucleotide sequences of reported gene. The antimicrobial susceptibility test showed that the four strains presented high resistance to carbapenems, cephalosporins and aminoglycosides (data not shown).

## Discussion

The rise of PCR, RT-PCR and other nucleic acid amplification technology greatly promoted the development of molecular biology. On-site diagnosis has been further facilitated as precise thermal cycler is not needed in isothermal nucleic acid amplification reaction.

The PSR method described in this study combines the advantage of PCR in which only one pair of primers is needed and isothermal amplification techniques such as RCR and 3SR. Primer design for PSR is very easy and convenient. We can use PCR primer design software (e.g., Primer 5, DNAMAN) to design a pair of common PCR primers. Then, all we need to do is to add the exogenous sequences (Nr and N) on the 5’ end of PCR primers. The Tm value of exogenous sequences was set 5 °C lower than the PCR sequences in order to ensure the conjugation of F and B to the target gene occurred earlier than the formation of spiral structure. In this study we abstracted the N and Nr sequences from a botanic gene to avoid nonspecific reaction with the target gene from microorganisms. Moreover, the current isothermal amplification methods either require an initial incubation at 95 °C (Loop-mediated isothermal amplification, Strand displacement amplification) or inclusion of a DNA helicase in the reaction mixture (Helicase-dependent amplification) to achieve the denaturation of Watson-Crick double strands. The PSR method does not need an initial denaturation step, the reaction proceeds as soon as the temperature reaches 61 °C to 65 °C.

Reaction components of PSR include Tris-HCl, KCl, (NH_4_)_2_SO_4_, Tween 20, MgSO_4_, dNTP, *Bst* DNA polymerase and Betaine which is a chemical destabilizing the DNA helix. These reagents can be mixed and stored under −20 °C before use, just like PCR MasterMix reagents. The reaction can be monitored through a real-time turbidimeter instrument or RT-PCR instrument with the addition of SYBR Greenı. Meanwhile, for visual detection purpose, aid from UV light or even the naked eye can directly recognize the result positive or negative.

Since the introduction of variable exogenous sequences (Nr and N), we could set restriction enzyme cutting sites on primer Ft and Bt artificially. After the completion of PSR reaction and digestion with the corresponding enzymes, the enzyme-digested product can be further used for sequencing and other molecular biology experiments. Subsequent experiments are in progress.

*bla*_NDM-1_ is a super antibiotic resistance gene emerged in recent years, with a total length of 813 bp. *Klebsiella pneumoniae*, *Escherichia coli* and other bacteria are always resistant to nearly all of the existing antibiotics after obtaining the *bla*_NDM-1_ gene, thereby the risk of nosocomial infection is greatly increased^16^. In this study, PSR was also applied to a clinical screening. Four strains containing *bla*_NDM-1_ with high antibiotic resistance were finally identified from clinical sputum samples, showing clinical significance of this method.

### Concluding remarks

The detection sensitivity of PSR method is as low as 6 cells per reaction within 45 minutes, and the positive results can be distinguished through simple color change, suggesting that this technique could also be applied in biosensor-based analytical instruments. PSR meets the guidelines proposed by the World Health Organization for developing diagnostic techniques, namely, ASSURED (affordable, sensitive, specific, user friendly, robust and rapid, equipment free and deliverable)^17^. The method provides a convenient and cost-effective alternative for clinical screening, on-site diagnosis and primary quarantine purposes.

## Methods

### Oligonucleotides and Enzymes

All oligonucleotides in this study were synthesized by Shenzhen BGI Biological Engineering Technology and Services Co. Ltd (Shenzhen, China). *Bst* DNA polymerase (large fragment) was purchased from New England Biolabs (Beijing, China).

### PSR amplification methods

The template target used in this study was the *E. coli* pGEX-NDM-BL21 containing *bla*_NDM-1_ gene constructed by our laboratory previously^18^. Bacterial strains (Table 1) were cultured in LB medium according to standard procedures. Then the genomic DNA was extracted using the Wizard Genomic DNA Purification Kit (Promega Co. USA).

The PSR reactions were carried out in a 25 μl reaction mixture containing the following components: 1.0 μl *Bst* DNA polymerase large fragment (New England Biolabs), 2.5 μl 10 × ThermolPol reaction buffer (New England Biolabs, including 20 mM Tris-HCl, 10 mM KCl, 10 mM (NH_4_)_2_SO_4_, 2 mM MgSO_4_, 0.1% Tween 20), 0.8 M Betaine (Sigma), 6 mM MgSO_4_, 1.4 mM each deoxynucleoside triphosphate. The amount of primers needed for one reaction was 1.6 μM for both Ft and Bt. Finally, an appropriate amount of DNA template was added to the reaction tube. The PSR reaction was carried out for 60 minutes at 65 °C, and the signal was acquired every 6 seconds using a real-time turbidimeter instrument.

Primers of PCR assay for *bla*_NDM-1_ was NDM-F (5’-ATGGAATTGCCCAATATTATGCA-3’, upstream primer) and NDM-R (5’-TCAGCGCAGCTTGTCGGCCATGC-3’, downstream primer). The PCR cycling parameters were: initial PCR activation, 95 °C for 5 min; amplification, 30 cycles of 95 °C for 30 s, 55 °C for 30 s, and 72 °C for 30 s; final extension, 72 °C for 10 min.

All experiments described here were replicated to ensure reproducibility.

## Additional Information

**How to cite this article**: Liu, W. *et al*. Polymerase Spiral Reaction (PSR): A novel isothermal nucleic acid amplification method. *Sci. Rep*. **5**, 12723; doi: 10.1038/srep12723 (2015).

## Figures and Tables

**Figure 1:** The schematic presentation and primer design of PSR method. (**A**): Schematic showing the mechanism of PSR. (**B**): Nucleotide sequence of *bla*_NDM-1_ (part) and locations of primers and restriction enzyme cutting sites are underlined. (**C**): Primer sequences of Ft and Bt targeting *bla*_NDM-1_ gene.

**Figure 2:** Sensitivity of serially diluted DNA quantitation by PSR amplification. (**A**): Isothermal amplification plot represents amplification products as observed through a real-time turbidimeter instrument every 6s at different concentrations of DNA. Data represents the mean of three replicates for each standard dilution. Amplification was performed at 65 °C for 60 min. (**B**): The standard curve obtained by plotting the value of crossing threshold (Ct) versus the concentration of CFU equivalents. 1, 6000 CFU; 2, 600 CFU; 3, 60 CFU; 4, 6 CFU; 5, 0.6 CFU; 6, 0.06 CFU; 7, negative control (double-distilled water).

**Figure 3:** (**A**): Gel electrophoresis results for PSR products of specificity experiment. (**B**): Visual results of PSR method under UV light. 1 to 6 are 10-fold serial dilution of the amplified product 6000, 600, 60, 6, 0.6, 0.06 CFU. 7 is the negative control (double-distilled water). Lane M is the 2000 bp molecular weight marker.

**Figure 4:** Gel electrophoresis results for PSR products prior and after restriction enzyme digestion. Lane1, PSR product that has been digested by Taq I; Lane 2 and 4, PSR product prior to digestion; Lane 3, PSR product that has been digested by Hinf I. Lane M is the 2000 bp molecular weight marker.

**Figure 5:** Specificity evaluation of PSR assay. (**A**): Real-time turbidimeter instrument recorded the PSR amplification plot of different clinical strains. Amplification was performed at 65 °C for 60 min. (**B**): PCR detection of *bla*_NDM-1_ in different strains. The product sequence is 813 bp. (**C**): Visual results of PSR method under UV light. 1, *Escherichia coli* pGEX-NDM-BL21; 2, *S. maltophilia* JKYJ-01; 3, *E. faecalis* PIJ; 4, *A. baumannii* H949; 5, *A. baumannii* B260; 6, *P. aeruginosa* D104; 7, *S. marcescens* SY-67; 8, *S. sonnei* 2531; 9, *S. flexneri* 4536; 10, *S. entericasero* type Paratyphi 86423; 11, enteroinvasive *E. coli* 44825; 12, enterotoxigenic *E. coli* 44824; 13, *V. carchariae* 5732; 14, *K. pneumoniae* 44824; 15, *V. parahaemolyticus* 5474; 16, negative control (distilled water).

**Table 1:** The clinical strains used for specificity test of PSR targeting *bla*_NDM-1_ gene.

Strains	Source
*S. maltophilia* JKYJ-01	Our microorganism center
*E. faecalis* PIJ	Our microorganism center
*A. baumannii* H949	Our microorganism center
*A. baumannii* B260	Our microorganism center
*P. aeruginosa* D104	Our microorganism center
*S. marcescens* SY-67	Our microorganism center
*S. sonnei* 2531	Our microorganism center
*S. flexneri* 4536	Our microorganism center
*S. entericaserotype Paratyphi* 86423	Our microorganism center
*enteroinvasive E. coli* 44825	Our microorganism center
*enterotoxigenic E. coli* 44824	Our microorganism center
*V. carchariae* 5732	Our microorganism center
*K. pneumoniae* 44824	Our microorganism center
*V. parahaemolyticus* 5474	Our microorganism center
